This article has been retracted.

# Involvement of Nrf2-Mediated Upregulation of Heme Oxygenase-1 in Mollugin-Induced Growth Inhibition and Apoptosis in Human Oral Cancer Cells

**DOI:** 10.1155/2013/210604

**Published:** 2013-05-02

**Authors:** Young-Man Lee, Q-Schick Auh, Deok-Won Lee, Jun-Yeol Kim, Ha-Jin Jung, Seung-Ho Lee, Eun-Cheol Kim

**Affiliations:** ^1^Department of Maxillofacial Tissue Regeneration and Research Center for Tooth & Periodontal Regeneration, School of Dentistry, Kyung Hee University, 1 Heogi-dong, Dongdaemun-gu, Seoul 130-701, Republic of Korea; ^2^Department of Oral Medicine, School of Dentistry, Kyung Hee University, Heogi-dong, Dongdaemun-gu, Seoul 130-701, Republic of Korea; ^3^Department of Oral and Maxillofacial Surgery, School of Dentistry, Kyung Hee University, Heogi-dong, Dongdaemun-gu, Seoul 130-701, Republic of Korea; ^4^College of Pharmacy, College of Pharmacy, Yeungnam University, Gyeongsan 712-749, Republic of Korea

## Abstract

Although previous studies have shown that mollugin, a bioactive phytochemical isolated from *Rubia cordifolia* L. (Rubiaceae), exhibits antitumor effects, its biological activity in oral cancer has not been reported. We thus investigated the effects and putative mechanism of apoptosis induced by mollugin in human oral squamous cell carcinoma cells (OSCCs). Results show that mollugin induces cell death in a dose-dependent manner in primary and metastatic OSCCs. Mollugin-induced cell death involved apoptosis, characterized by the appearance of nuclear shrinkage, flow cytometric analysis of sub-G_1_ phase arrest, and annexin V-FITC and propidium iodide staining. Western blot analysis and RT-PCR revealed that mollugin suppressed activation of NF-**κ**B and NF-**κ**B-dependent gene products involved in antiapoptosis (Bcl-2 and Bcl-xl), invasion (MMP-9 and ICAM-1), and angiogenesis (FGF-2 and VEGF). Furthermore, mollugin induced the activation of p38, ERK, and JNK and the expression of heme oxygenase-1 (HO-1) and nuclear factor E2–related factor 2 (Nrf2). Mollugin-induced growth inhibition and apoptosis of HO-1 were reversed by an HO-1 inhibitor and Nrf2 siRNA. Collectively, this is the first report to demonstrate the effectiveness of mollugin as a candidate for a chemotherapeutic agent in OSCCs via the upregulation of the HO-1 and Nrf2 pathways and the downregulation of NF-**κ**B.

## 1. Introduction

Oral squamous cell carcinoma (OSCC) represents the fifth most common cancer worldwide and is a significant cause of cancer morbidity and mortality. Each year, approximately 300,000 new cases are diagnosed with only a 50% survival rate over 5 years. Common treatments, including surgery, radiation therapy, and chemotherapy, have very low success rates [1]. Two of the most frequently used chemotherapeutic drugs, 5-fluorouracil and cisplatin, cause side effects such as bone marrow suppression, gastrointestinal toxicity, and renal damage, which remain problems that need to be resolved [2]. To overcome such side effects and limitations, the direction of present research into novel antitumor agents has turned to natural products, especially plants used in traditional medicine [3]. Previously, we demonstrated that highly purified sulfur [4] and herbal medicines, such as *Caesalpinia sappan* [5], *Coptidis rhizoma *[6], and verticinone [7], exerted antitumor effects on oral cancer cells* in vitro.* Moreover, we showed that a single compound isolated from *Caesalpinia sappan* heartwood, isoliquiritigenin 2′-methyl ether (ILME), had antioral cancer effects involving mitogen-activated protein kinases (MAPKs) and the nuclear factor-*κ*B (NF-*κ*B) pathway [8]. In addition, we reported that a flavonoid extracted from *Caesalpinia sappan*, sappanchalcone, suppressed oral cancer cell growth and induced apoptosis through activation of p53-dependent mitochondrial MAPK and NF-*κ*B signaling [9].

The roots of *Rubia cordifolia* L. have been widely used as a traditional herbal medicine in Korea to treat cough, bladder and kidney stones, joint inflammation, uterine hemorrhage, and uteritis [10]. In addition, this plant has been used in traditional Chinese medicine for the treatment of arthritis, dysmenorrheal, hematorrhea, hemostasis, and psoriasis [11, 12]. Among the bioactive components from *Rubia cordifolia*, mollugin (C_17_H_16_O_4_; methyl 2,2-dimethyl-6-hydroxy-*2H*-naphtho[1,2-*b*]pyran-5-carboxylate) has been reported to have antitumor and anti-inflammatory activities, and neuroprotective and apoptotic effects [13–16]. A recent study demonstrated that mollugin induced apoptosis through endoplasmic reticulum stress-mediated activation of c-Jun N-terminal kinase (JNK) and the mitochondria-dependent caspase cascade, regulated by Bcl-xL in human Jurkat T cells [14]. Moreover, mollugin inhibited proliferation and induced apoptosis by suppressing fatty acid synthase in HER2-overexpressing human breast and ovarian cancer cells [17].

Heme oxygenase-1 (HO-1) is an inducible cytoprotective enzyme that catalyzes the initial rate-limiting reaction in heme catabolism. Previously, we reported that the HO-1 pathway plays a key role in the adaptation of cells to stressful conditions and the recovery of dental pulp cells and periodontal ligament cells from injury [18–20]. Despite its cytoprotective properties, recent evidence suggests a role for HO-1 in promoting cancer [21]. HO-1 is overexpressed in various types of cancer and is further induced by radiation and chemotherapy [22, 23]. Regarding the mechanisms of HO-1 induction, several studies have suggested the involvement of MAPK and NF-*κ*B pathways, as well as nuclear factor erythroid 2–related factor 2 (Nrf2) [18, 24]. However, the precise cellular mechanisms of mollugin on OSCCs are not completely understood.

The aim of this study was to investigate the chemotherapeutic effect of mollugin on human primary and metastatic OSCCs *in vitro*. In addition, we further explored whether the effect of mollugin is related to Nrf2 activation and HO-1 expression.

## 2. Materials and Methods 

### 2.1. Reagents

Mollugin was isolated from root of heartwood of *Rubia cordifolia* L. as described previously [13]. Antibody against NF-*κ*B p65, I*κ*B, Nrf2, Bcl-xL, Bcl-2, p53, p21, or phosphorylated isoforms of I*κ*B and horseradish peroxidase-conjugated secondary antibodies were purchased from Santa Cruz Biotechnology (Delaware Avenue, CA). ERK, JNK, p38 or phosphorylation of ERK, JNK, and p38 were purchased from Cell signaling, Inc. (Beverly, MA). Dulbecco's modified Eagle's medium (DMEM), fetal bovine serum (FBS), and other tissue culture reagents were purchased from Gibco BRL (Grand Island, NY). All other chemicals were obtained from Sigma (St. Louis, MO), unless indicated otherwise. 

### 2.2. Cell Culture

The cell line HNSCC4 (HN4), from a primary OSCCs, and cell line HNSCC12 (HN12), from a metastatic carcinoma of the OSCCs [25], were derived in the laboratory of Dr. John F. Ensley (Wayne State University). Cells were cultured in DMEM supplemented with 10% FBS, 100 U/mL penicillin, and 100 *μ*g/mL streptomycin in a humidified atmosphere of 5% CO_2_ at 37°C. Cells were dissociated with 0.25% trypsin just before transferring for experiments and counted using a hemocytometer.

Human keratinocyte cell line HaCaT (nontransformed human cell line) were incubated in DMEM supplemented with 10% FBS, 1 mM sodium pyruvate, 50 *μ*g/mL streptomycin, and 50 *μ*g/mL penicillin at 37°C in 5% CO_2_. Human gingival fibroblasts (HGFs) cell line by transfection with the E6/E7 open reading frames of HPV type 16 was cultured according to the following protocol, as reported by our study [26]. Briefly, HGFs were cultured in DMEM supplemented with 10% FBS, 100 U/mL penicillin, and 100 *μ*g/mL streptomycin in a humidified atmosphere of 5% CO_2_ at 37°C.

### 2.3. Antiproliferative Assay

Cell viability was determined by 3-(4,5-Dimethylthiazol-2-yl)-2,5-diphenyltetrazolium bromide (MTT) assay. Briefly, cells were seeded in flat-bottomed 96-well plates, at 1 × 10^5^ cell/well 24 h prior to treatment. The cells were treated for various lengths of time with the agents indicated. Then 25 *μ*L of 5 mg/mL MTT was added to each well. After 4 h incubation at 37°C, 100 *μ*L of lysing buffer was added. The buffer consisted of 20% w/v of sodium dodecyl sulfate in 0.1% of HCl solution. The plates were incubated for a further analysis on an ELISA reader at 570 nm. The same experiment was repeated in three separate cultures, and the data were presented as the means ± SD of five observations.

### 2.4. Flow Cytometry

#### 2.4.1. Propidium Iodide (PI) Staining

Cells were seeded at 5 × 10^5^cells/well in six-well plates. After 24 h, cells were treated with mollugin the 3 days. After treatment, cells were harvested and pelleted by centrifugation (400 ×g, 4°C, 5 min). The cells were fixed with cold 75% ethanol for 24 h and then stained with PI solution, consisting of 45 mg/mL PI, 10 mg/mL RNase A, and 0.1% Triton X-100. After incubation in the dark at 4°C for 1 h, fluorescence-activated cells were sorted using the FACScan flow cytometer, and the data were analyzed using Cellfit Analysis Software. 

### 2.5. Fluorescein-Isothiocyanate-(FITC-) Annexin V and Propidium Iodide (PI) Double Staining

Cells (5 × 10^5^) were seeded in 6-well plates, incubated for 24 h, and then treated with or without mollugin, and the incubation was continued for 3 days. After treatment, the cell pellet was prepared in a FACStar tube containing annexin V-FITC solution and incubated in 5% CO_2_ at 37°C. The PI solution (without NP 40) was then added, and the ratio of PI-positive and annexin V-positive cells was measured using the flow cytometer. 

### 2.6. Morphological Analysis of Apoptosis by Staining with 4′,6-Diamino-2-Phenylindole Dihydrochloride (DAPI)

To confirm that the nuclei underwent morphological changes, the cells were cultured in 60 mm dishes overnight and then washed twice in DMEM. The cells were then treated with mollugin and fixed in 4% paraformaldehyde, after which they were incubated in 1 *μ*g/mL DAPI solution for 30 min in the dark. The cells were then examined using a fluorescence microscope (Zeiss, Oberköchen, Germany). 

### 2.7. Western Blot Analysis

Western blot analysis was performed by lysing cells in 20 mM Tris-HCl buffer (pH 7.4) containing protease inhibitor mixture (0.1 mM phenylmethanesulfonyl fluoride, 5 mg/mL aprotinin, 5 mg/mL pepstatin A, and 1 mg/mL chymostatin). Protein concentration was determined using the Lowry protein assay kit (P5626; Sigma). An equal amount of protein for each sample was resolved using 7% or 12% sodium dodecyl sulfate-polyacrylamide gel electrophoresis (SDS-PAGE) and then electrophoretically transferred onto a Hybond-enhanced chemiluminescence (ECL) nitrocellulose membrane (Bio-Rad, Hercules, CA). The membrane was blocked with 5% skim milk and sequentially incubated with primary antibody (Santa Cruz Biotechnology) and horseradish peroxidase-conjugated secondary antibody followed by ECL detection (Amersham Pharmacia Biotech, Piscataway, NJ).

### 2.8. Isolation of RNA and RT-PCR

Total RNA was isolated using the TRIzol reagent (Invitrogen, Carlsbad, CA, USA) according to the manufacturer's instructions. It was then reverse-transcribed using AccuPower RT premix (Bioneer, Daejeon, Korea). The PCR amplification of the resulting cDNA samples was performed using a GeneAmp PCR System 2400 thermal cycler (PerkinElmer, Wellesley, MA, USA). The primers information is summarized in Table 1. The following PCR conditions were used: 34 cycles of denaturation at 95°C for 30 s, primer annealing at 60°C for 30 s, and extension at 72°C for 30 s. The PCR products were resolved on 1-2% agarose gels and stained with ethidium bromide.

### 2.9. HO-1 and Nrf2 siRNA Transfection

The target sequence for human HO-1 siRNA was 5′-AACUUUCAGAAGGGCCAGGUGTT-3′ (forward) and 5′-CACCUGGCCCUUCUGAAAGUUTT-3′ (reverse). Transfection of Nrf2 siRNA was performed using the target sequence 5′-AAGAGUAUGAGCUGGAAAAACTT-3′ (forward) and 5′-GUUUUUCCAGCUCAUACUCUUTT-3′ (reverse). Cells were transfected with siRNA using Lipofectamine RNAiMAX (Invitrogen) according to the manufacture's instruction. Silencer Negative Control siRNA (Invitrogen) was introduced into cells by the same method. Following transfection, cells were cultured in six-well plates at 37°C until required.

### 2.10. Statistical Analysis

Data are expressed as the mean ± standard deviation. Statistical comparisons of the results were made using analysis of variance (ANOVA). Significant differences (*P* < 0.05) between the means of control and sulfur-treated cells were analyzed using Dunnett's test. 

## 3. Results

### 3.1. Effect of Mollugin on HN4 and HN12 Cell Viability

To investigate the effect of mollugin on the proliferation of human OSCCs, the MTT assay was used. As shown in Figure 1, mollugin inhibited cellular proliferation in a dose- and time-dependent manner. Moreover, mollugin displayed higher cytotoxicity in primary OSCC HN4 cells compared with metastatic OSCC HN12 cells, although the overall trend of the effects of mollugin on HN4 and HN12 cells was similar. Furthermore, we tested whether mollugin has any toxic effect on nonneoplastic human skin keratinocytes (HaCaT) and gingival fibroblasts (GF). Interestingly, we did not find significant cytotoxicity or cell death by mollugin on HaCaT and GF (Figures 1(c) and 1(d)).

### 3.2. Effect of Mollugin on HN4 and HN12 Cell Apoptosis

To determine whether the cause of cell death was apoptosis, HN4 and HN12 cells were exposed to 40 *μ*M mollugin for 3 days. This concentration was used because it reproducibly induced 50% growth inhibition in HN4 and HN12 cells cultured for 3 days. Cell nuclei were stained with 4′,6-diamidino-2-phenylindole (DAPI), a fluorescent DNA-binding dye (Figure 2(a)). DAPI staining showed that the control nuclei were large and round without condensation or fragmentation, whereas most of the nuclei of mollugin-treated cells were condensed and fragmented, as is typical during apoptosis. The onset of apoptotic cell death by mollugin was confirmed by flow cytometry of HN4 and HN12 cells (Figure 2(b)). Without treatment, only 3.88% HN4 and 2.80% HN12 cells were in the sub-G_1_ region; however, mollugin treatment increased the proportions of cells in the sub-G_1_ region to 20.26% and 31.46%, respectively. To determine whether the growth inhibitory effect of mollugin is associated with cell death, annexin V-propidium iodide (PI) double staining of HN4 and HN12 cells and flow cytometry was performed (Figure 2(c)). Treatment of cells with mollugin for 3 days increased the number of annexin V^+^/PI^+^ stained cells. These results demonstrate that the inhibition of cell growth by mollugin was caused by the induction of apoptosis.

### 3.3. Effect of Mollugin on NF-*κ*B Activation and Expression of NF-*κ*B-Regulated Genes

Since NF-*κ*B transcription factors and their upstream activating molecules are attractive targets for cancer therapeutics, we evaluated the effect of mollugin on NF-*κ*B activation by measuring the phosphorylation and degradation of I*κ*B*α* and NF-*κ*B p65. As shown in Figure 3(a), treatment of HN4 and HN12 cells with mollugin decreased the steady-state levels of phosphorylated I*κ*B*α* and nuclear NF-*κ*B p65.

To clarify the molecular mechanism by which mollugin induces apoptosis in primary and metastatic OSCCs, we determined the levels of NF-*κ*B-regulated gene products involved in apoptosis and antiapoptosis (Figure 3(b)). Mollugin treatment upregulated p53 and p21 expression in both HN4 and HN12 cells in a dose-dependent manner. In contrast, the expression of antiapoptotic Bcl-2 and Bcl-xl proteins was dose-dependently reduced by mollugin treatment in HN4 and HN12 cells. Next, we investigated whether mollugin could modulate levels of NF-*κ*B-regulated gene products involved in invasion (ICAM-1 and MMP-9) and angiogenesis (VEGF and FGF-2) of OSCCs. The results show that mollugin downregulated the expression of NF-*κ*B-regulated gene products, including MMP-9, ICAM-1, VEGF, and FGF-2 mRNA in a dose-dependent manner (Figure 3(c)).

### 3.4. Effect of Mollugin on MAPK and Nrf2 Activation

To clarify the mechanism underlying the apoptosis, we assessed the effect of mollugin on Nrf2 and NF-*κ*B upstream pathways. Treatment with mollugin (40 *μ*M) increased levels of phosphorylated (activated) ERK, p38, and JNK; the phosphorylated proteins were easily detectable by Western blot after 30 or 60 min. In contrast, mollugin did not affect total p38, ERK, or JNK levels (Figure 4(a)). 

Since the stress response element/Nrf2 transcription factor pathway is important for HO-1 expression [23], we next determined whether Nrf2 signaling is involved in mollugin-induced HO-1 expression and apoptosis. Initially, Nrf2 activation was assessed by the accumulation of Nrf2 in the nucleus. Treatment with mollugin resulted in an accumulation of Nrf2 in the nucleus in primary and metastatic OSCCs (Figure 4(b)).

To determine whether mollugin induces expression of antioxidant genes, HO-1 expression in oral cancer cells and the change in the pattern of HO-1 expression were evaluated. HO-1 protein expression in primary and metastatic OSCCs increased following mollugin treatment in a time-dependent manner (Figure 4(c)).

To confirm the involvement of MAPK pathways in the mollugin-driven activation of NF-*κ*B and Nrf2, inhibitors of ERK (PD98059), JNK (SP6100126), and p38 (SB203580) MAPK signaling were used. Mollugin-induced NF-*κ*B, Nrf2, and HO-1 expression was effectively inhibited by PD98059, SP600126, and SB203580 (Figure 4(d)), suggesting that p38, ERK1/2, and JNK play important roles in activating NF-*κ*B, Nrf2, and HO-1 in HN4 and HN12 cells.

### 3.5. Involvement of the HO-1 Pathway in Mollugin-Induced Apoptosis

To examine the cytotoxic potential of tin protoporphyrin (SnPP), an HO-1 inhibitor, its effect on viability was initially measured by the MTT assay (Figure 5(a)). Although, 10 or 20 *μ*M SnPP had no cytotoxicity effect for 3 h, we found that SnPP exhibited slight cytotoxicity on HN4 and HN12 cells at 16 h. Based on these findings, we chose to use SnPP for 3 h. 

To determine whether the induction of HO-1 plays a role in mollugin-induced growth inhibition and apoptosis in OSCCs, cells were treated with SnPP, an HO-1 inhibitor, for 3 h before incubation with mollugin for 3 days. MTT assays showed that mollugin-induced cytotoxicity and apoptosis in HN4 and HN12 cells were dose-dependently reversed by pretreatment with SnPP (Figures 5(a) and 5(b)). In addition, SnPP treatment abolished the induction of p53 and p21^WAF1/CIP1^ expression by mollugin, but reversed the expression of Bcl-2 and Bcl-xl (Figure 5(c)).

 Additionally, we used a siRNA-expressing plasmid to induce HO-1 gene silencing. HN4 and HN12 cells were transfected with an HO-1-targeting siRNA expression vector (Figure 6). The siRNA approach resulted in high silencing efficacies for HO-1, which was confirmed by Western blot analysis (Figure 6(c)). Silencing of HO-1 significantly attenuated mollugin-induced cytotoxicity (Figure 6(a)) and apoptosis (Figure 6(b)). Moreover HO-1 RNA blocked mollugin-induced Nrf2, p53, and p21 upregulation as well as Bcl-2 and Bcl-xl downregulation (Figure 6(c)).

### 3.6. Involvement of the Nrf2 Pathway in Mollugin-Induced HO-1 Induction and Apoptosis

To investigate whether mollugin-induced apoptosis and HO-1 expression were mediated by Nrf2 activation, a specific small interfering RNA (siRNA) against Nrf2 was used. As shown in Figure 7(c), transfection with Nrf2 siRNA for 5 h in HN4 and HN12 cells blocked mollugin-induced HO-1 and Nrf2 expression. However, Nrf2 siRNA did not affect the mollugin-induced p65 expression. Transfection with Nrf2 siRNA inhibited mollugin-induced cytotoxicity and apoptosis in HN4 and HN12 cells (Figures 7(a) and 7(b)). Moreover, transfection with Nrf2 siRNA in HN4 and HN12 cells reduced mollugin-induced apoptosis proteins (p53 and p21), but reversed antiapoptosis proteins (Bcl-2 and Bcl-xl) (Figure 7(c)).

## 4. Discussion

This study is to our knowledge the first to demonstrate that mollugin directly induces growth inhibition and apoptosis in primary and metastatic OSCCs and to address the molecular basis of this effect. 

With regard to antitumor activity, mollugin has been shown to exert cytotoxic effects on human colon cancer (Col2) cells (IC_50_ = 12.3 *μ*M; [11]), human liver carcinoma (HepG2) cells (IC_50_ value = 60.2 *μ*M; [10]), and basal HER2-expressing human breast cancer cells (IC_50_ value = 58 *μ*M; [17]). In the present study, we found that mollugin (10–80 *μ*M) resulted in significant growth inhibition, with an average IC_50_ value of 46.3 *μ*M in metastatic OSCCs (HN12) and 43.9 *μ*M in primary OSCCs (HN4) after 3 days. These antiproliferative properties of mollugin are consistent with previous reports in human acute leukemia Jurkat T cells [14] and HER2-overexpressing breast and ovarian cancer cell lines [17]. Moreover, we demonstrated that mollugin induced OSCC cell death by triggering apoptosis due to the presence of several apoptotic characteristics, including sub-G_1_ phase accumulation, increase in annexin^+^/PI^+^ cells, and DNA fragmentation. 

NF-*κ*B signaling is a ubiquitous pathway in cell proliferation, survival, and apoptosis. Normally, NF-*κ*B proteins are inhibited by binding to I*κ*B proteins in the cytoplasm. Stress factors cause degradation of I*κ*B proteins through the ubiquitin-proteosomal pathway, and NF-*κ*B is released to bind to the DNA of promoter regions of specific genes that increases their transcription rate [27, 28]. To explore the mechanism underlying mollugin-induced apoptosis in OSCCs, we examined NF-*κ*B activation. In agreement with previous findings that mollugin suppressed NF-*κ*B activation in HER2-overexpressing SK-BR-3 breast cancer cells [17], our results indicate that mollugin significantly inhibited NF-*κ*B activation by reducing the level of phospho-I*κ*B*α*, leading to blockage of the I*κ*B*α* pathway in NF-*κ*B activation in OSCCs. In addition, it was reported that mollugin significantly suppressed TNF-*α*-induced NF-*κ*B transcriptional activation in HT-29 human colonic epithelial cells [13]. 

Genes involved in the proliferation, apoptosis, antiapoptosis, angiogenesis, and metastasis of cancer are regulated by NF-*κ*B [29]. Constitutive activation of NF-*κ*B negatively regulates the proapoptotic functions of p53 by inducing the expression of an array of antiapoptotic genes, including Bcl-2 and Bcl-xL [30]. In our study, treatment with mollugin induced the downregulation of antiapoptotic Bcl-2 and Bcl-xL levels as well as the upregulation of apoptotic p53 and p21 levels in OSCCs. Another hallmark of OSCC behavior is their propensity for local invasion and metastasis. MMP-9 is frequently overexpressed in OSCCs and is dependent upon NF-*κ*B for expression [31]. Adhesion molecules such as ICAM-1 are regulated by NF-*κ*B and are essential for the adhesion of tumor cells to endothelial cells and thus mediate tumor cell metastasis [32]. Angiogenesis is important for tumor growth and progression. The development of angiogenesis is stimulated by cytokines and growth factors, and the expression of these cytokines and growth factors is correlated with the pathological neovascularization circumstances. Among these angiogenic factors, VEGF and FGF-2 are important angiogenic factors and essential for cancers [33]. In this study, we found that mollugin inhibited the expression of NF-*κ*B-regulated gene products involved in invasion (MMP-9 and ICAM-1) and angiogenesis (FGF-2 and VEGF). Thus, our results demonstrate that mollugin inhibits NF-*κ*B, leading to suppression of proliferation, invasion, and angiogenesis in OSCCs.

The MAPKs are proline-directed Ser/Thr protein kinases that regulate many cellular processes, including cell proliferation and death. JNK and p38 are activated by cellular stress and are associated with apoptosis [34]. The involvement of ERK in the induction of apoptosis by quercetin, resveratrol, and taxol has been reported [35, 36]. In the present study, phosphorylation of p38, ERK, and JNK was detected in mollugin-treated OSCCs, which is consistent with our previous reports that sappanchalcone may exert its effect on OSCCs through p38, ERK, and JNK activation [9]. Therefore, NF-*κ*B regulation downstream of the MAPK (ERK1/2, p38, and JNK) pathways may be involved in mollugin-induced apoptosis in OSCCs. However, mollugin activated p38 MAPK in hippocampal and microglial cells [15] and ERK in HER2-overexpressing breast cancer cells [17]. Therefore, MAPK can be differentially activated, and its involvement in apoptosis is highly context and model dependent. 

The role of HO-1 in tumor development is still not understood completely. Some recent reports demonstrate discordant or even completely contrasting results. Nevertheless, accumulating evidence indicates that HO-1 is expressed or overexpressed in a wide variety of human tumors and plays a critical role in the progression of neoplastic diseases [37]. For example, it has been shown that increased expression of HO-1 is associated with a higher rate of proliferation of various tumor cells [37, 38], although opposite effects have been observed in breast cancer cells [39]. Furthermore, the increased basal level of HO-1 expression in tumor cells can be further elevated by chemotherapeutics or phytochemicals, such as curcumin, carnosol, and ILME [8, 22, 23]. Our results show that mollugin upregulated HO-1 expression in a time- and dose-dependent manner (data not shown), consistent with results in hippocampal and microglial cells [15]. We found that growth inhibition and apoptosis of OSCCs by mollugin was reversed in the presence of an HO-1 inhibitor. In addition, mollugin induced downregulation of antiapoptotic Bcl-2 and Bcl-xL levels, while upregulation of apoptotic p53 and p21 levels was reversed by SnPP in a dose-dependent manner. These results suggest that the growth inhibition and apoptosis-inducing effect of mollugin is mediated via HO-1 expression. 

Regarding HO-1, Nrf-2 is a relatively well-known transcription factor [40]. In response to diverse HO-1 inducers, Nrf2 translocates from the cytosol to the nucleus where it binds to the antioxidant response element in the promoter region of the HO-1 gene [41]. In our study, mollugin also induced the translocation of Nrf-2 into the nucleus, as evidenced by Western blot. Furthermore, the results of this study demonstrate a correlation between apoptotic gene upregulation and the suppression of antiapoptotic genes of OSCCs to undergo mollugin-induced growth inhibition and apoptosis when Nrf-2 is knocked down. Based on these observations, it is reasonable to conclude that Nrf2 activation mediates mollugin-induced growth inhibition and apoptosis in OSCCs. 

Redox-sensitive transcription factor (NF-*κ*B, AP-1, and Nrf2) pathways are known to be important molecular targets in chemoprevention. Activation of Nrf2 and NF-*κ*B involves regulation of protein kinases, which may induce their nuclear translocation [42]. It was previously shown that mollugin induced apoptosis via JNK in human Jurkat T cells [14]. In this regard, specific protein kinase inhibitors of PI3 K and ERK repressed Nrf2 phosphorylation and nuclear translocation of Nrf2 and NF-*κ*B in HepG2 cells, as previously reported in different cell types [43, 44]. The present results also suggest that the MAPK pathway plays a role in the mollugin-induced nuclear translocation of Nrf2 and NF-*κ*B in HN4 and HN12 cells. A variety of anticarcinogenic phytochemicals suppress NF-*κ*B signalling and activate the Nrf2-ARE pathway [45], suggesting that the suppression of NF-*κ*B signalling and the activation of the Nrf2-ARE pathway may crosstalk with each other. Indeed, inhibition of NF-*κ*B activation by phospholipid hydroperoxide glutathione peroxidase and 15-lipoxygenase is concomitant to upregulation of HO-1, probably via Nrf2 activation [46]. Thus, the findings support that the participation of NF-*κ*B p65 in the negative regulation of Nrf2-ARE signalling, providing a new insight into a possible role of NF-*κ*B in suppressing the expression of anti-inflammatory or antitumour genes [47]. Our results suggest that MAPK singnaling event mediates the link between NF-*κ*B and Nrf2. Although the NF-*κ*B pathway was inhibited by mollugin exposure, Nrf2 siRNA did not seem to participate in the translocation of NF-*κ*B, suggesting that NF-*κ*B and Nrf2 pathways might act in parallel in our *in vitro* model. A summary of our results is shown in Figure 8. 

Colectivelly, our results demonstrate for the first time that mollugin inhibits cell growth and induces apoptosis in OSCCs through the NF-*κ*B/MAPK/Nrf2/HO-1 signaling pathway. Therefore, mollugin may have potential as a chemotherapeutic agent for OSCCs. The activities of mollugin against multiple antitumor targets should be studied intensively for further clinical application either as a natural agent alone or in combination with other commonly used chemotherapeutics. Further investigation of mollugin in animal models of OSCCS will contribute to additional understanding of its *in vivo* activity toward malignant cells and its potential toxicity toward normal tissues.

## Figures and Tables

**Figure 1:** Effects of mollugin on cell viability in primary (HN4, (a)), metastatic oral cancer cells (HN12, (b)), skin keratinocytes (HaCaT, (c)), and gingival fibroblasts (d) as measured by MTT assay. *Statistically significant difference as compared to control, *P* < 0.05. The same experiment was repeated in three separate cultures, and the data were presented as the means ± SD of five observations.

**Figure 2:** Confirmation of mollugin-induced apoptosis by DAPI staining (a), cell cycle analysis (b), and annexin V-PI staining (c) in OSCCs. Cells were incubated with 40 *μ*M mollugin for 3 days. Data are presented as mean ± SD from triplicate determinations (b, c). Results are representative from three independent experiments (a)–(c).

**Figure 3:** Effects of mollugin on activation of NF-*κ*B (a), and expression of NF-*κ*B-regulated gene products involved in apoptosis and antiapoptosis (b), metastasis, and angiogenesis (c) in OSCCs. Cells were treated with 40 *μ*M mollugin for indicated times (a) or 3 days (b, c). The figure is representative of 3 independent experiments.

**Figure 4:** Effect of mollugin on phosphorylation of MAPK (a), activation of Nrf2 (b), and expression of HO-1 (c) in OSCCs. Effects of MAP kinase inhibitors on mollugin-induced activation of NF-*κ*B, Nrf2, and HO-1 (d). Cells were treated with 40 *μ*M mollugin for indicated times (a)–(c). Cells were pretreated with the p38 inhibitor SB203580 (20 *μ*M/L), the ERK inhibitor PD98059 (20 *μ*M/L), or the JNK inhibitor SP600125 (20 *μ*M/L) for 1 hour and treated with 40 *μ*M mollugin for 30 min (MAPK, Nrf2, and NF-*κ*B) or 3 days (HO-1). The results are representative of three independent experiments.

**Figure 5:** Effects of HO-1 inhibitor (SnPP) on cytotoxicity (a), mollugin-induced growth inhibition (b), apoptosis (c), and apoptosis-related proteins expression (d) in OSCCs. Cells were pretreated with SnPP for 3 h and treated for 3 days with mollugin (b)–(d). Cell viability was examined by MTT assay (a), and apoptosis was examined by flow cytometry (b), respectively. The same experiment was repeated in three separate cultures, and the data were presented as the means ± SD of five observations (a, b). Data are presented as mean values from triplicate determinations (c). Western data show one representative result of three independent experiments (d). *Statistically significant difference as compared to control, *P* < 0.05. ^#^Statistically significant difference as compared to mollugin, *P* < 0.05.

**Figure 6:** Effects of HO-1 siRNA on mollugin-induced growth inhibition (a), apoptosis (b), and apoptosis-related proteins expression (c) in OSCCs. Cells were pretreated with HO siRNA (30 nM) for 5 h and treated for 3 days with mollugin (a)–(c). Cell viability was examined by MTT assay (a), and apoptosis was examined by flow cytometry (b), respectively. The same experiment was repeated in three separate cultures, and the data were presented as the means ± SD of five observations (a). Data are presented as mean values from triplicate determinations (b). Western data show one representative result of three independent experiments (c). *Statistically significant difference as compared to control, *P* < 0.05. ^#^Statistically significant difference as compared to mollugin, *P* < 0.05.

**Figure 7:** Effect of Nrf2 siRNA on mollugin-induced growth inhibition (a), apoptosis (b), and apoptosis-related proteins expression (c). Cells were treated with 40 *μ*M mollugin for indicated times (a). Cells were pretreated with Nrf2 siRNA (250 nM) for 5 h and treated for 3 days with mollugin 40 *μ*m (a)–(c). *Statistically significant difference as compared to control, *P* < 0.05. ^#^Statistically significant difference as compared to mollugin, *P* < 0.05. Data are representative of 3 independent experiments.

**Figure 8:** Schematic diagram illustrating the Nrf2 pathway and other signaling pathways triggered by exposure to mollugin in in OSCCs. Mollugin treatment leads to the activation of the cellular stress-dependent signaling pathways mediated by MAPK activation (ERK, JNK, and p38) and subsequent transcription factor activation (NF-*κ*B and Nrf2). Ultimately, these transcription factors result in altered gene expression to produce cytoprotective gene HO-1, allowing lead to apoptosis.

**Table 1:** Reverse transcriptase-polymerase chain reaction primers.

Gene	Sequence 5′-3′	Size
MMP-9	Forward: GTTGGGGAGGGCTGTCCGTGA	911 bp
	Reverse: CGTGGCGCTATCCAGCTCACC	
ICAM-1	Forward: CGCCCGATTGCTTTAGCTTG	320 bp
	Reverse: CGACTCACCTGGGAACAGAG	
VEGF	Forward: TCAAGGTTGGCGGAAGTGAGG	443 bp
	Reverse: CCCTTGCATCAGTAGGCTTCA	
FGF2	Forward: GCCTCATTTCCATTTCGTGG	224 bp
	Reverse: CGGGGGTACTGGTTTACAG	
*β*-actin	Forward: CATGGATGATGATATCGCCGC	319 bp
	Reverse: ACATGATCTGGGTCATCTTCT	
